# Effectiveness of Super-selective Embolization for Parasagittal Meningiomas and Its Effect on the Level of Inflammatory Factors

This article has been retracted.

**DOI:** 10.1155/2022/2466007

**Published:** 2022-08-01

**Authors:** Zhaoke Zheng, Linwei Jia, Peihua Zhang, Yaohui Tian, Xi Chen

**Affiliations:** Second Department of Neurosurgery, Cangzhou Central Hospital, Cangzhou, China

## Abstract

**Objective:**

To evaluate the effectiveness of super-selective embolization for parasagittal meningiomas and its effect on the level of inflammatory factors.

**Methods:**

A total of 48 patients with parasagittal meningiomas diagnosed and treated in our hospital from September 2018 to March 2020 were randomly included and assigned to receive meningioma resection (control group) or meningioma resection plus super-selective embolization (study group), with 24 patients in each group. Outcome measures included clinical indices, tumor resection outcome, inflammatory factor levels, and follow-up results.

**Results:**

Patients in the study group had shorter operative time and less intraoperative bleeding volume than those in the control group (*P* < 0.05). The study group had more patients with Simpson I resection (87.50%) than the control group (62.50%) (*P* < 0.05). There was no statistically significant difference in the levels of inflammatory factors between the two groups of patients before treatment (*P* > 0.05). After treatment, the levels of interleukin (IL)-6, tumor necrosis factor (TNF)-*α*, and hypersensitive C-reactive protein (hs-CRP) in patients in the study group were significantly lower than those of the control group. The results of the three-month follow-up showed that one patient in the study group was reoperated for tumor recurrence and there was no death record, while three patients in the control group were reoperated for tumor recurrence and one patient died. The difference in the recurrence and mortality between the two groups did not come up to the statistical standard (*P* > 0.05).

**Conclusion:**

Super-selective embolization for parasagittal meningiomas contributes to reducing intraoperative bleeding, effectively improving tumor resection and surgical safety, and lowering inflammatory factor levels. Further trials are, however, required before clinical promotion.

## 1. Introduction

Meningioma [1] is the most common type of primary intracranial tumor of the central nervous system, accounting for about one-third of all tumors of the central nervous system. It is a brain tumor originating from the meninges and arachnoid capillary cells, mostly with benign development [2]. According to relevant epidemiological statistics, the annual prevalence of meningioma is 1∼8/100000, ranking the second-highest among intracranial tumors. Its incidence increases with age and peaks at the age of 45 years, with a gender ratio of male to female being 1 : 2 [3]. Meningioma is usually asymptomatic in the early stage and mainly occurs in the convex surface of the cerebral hemisphere, skull base, and paracellular area, and about 50% is located near the sagittal sinus, more common in the convex surface of the brain next to the sickle, followed by the pterygoid crest, cerebellar nodes, odor, cerebellar pontocerebellar angle, and the canopy [4]. Parasagittal meningiomas [5] are usually adherent to the falx cerebri, and about 1/4 are bilateral lesions [6, 7]. Epilepsy is its initial symptom, with partial or grand mal seizures, and psychiatric disorders manifest as dementia and emotional indifference. In addition, patients are prone to personality changes, and paragangliomas located in the occipital lobe can cause visual field disturbances [8].

The clinical treatment is mainly surgical resection supplemented with radiation therapy [9]. However, due to the complexity and severity of the disease, lateral rupture of the sagittal sinus may occur during surgery may result in hemorrhage, or the tumor may form adhesion with the sagittal buccal cavity wall, resulting in incomplete removal of the tumor and postoperative recurrence. [10]. Thus, patients are predisposed to postoperative complications such as hemiparesis and aphasia. Traditional Chinese medicine believes that the excess or deficiency of the seven emotions can lead to abnormal qi and blood circulation in the body and dysfunction of the viscera. The occurrence and development of some cancers are mostly related to emotional insufficiency. The formation of brain tumors is mainly caused by phlegm blocking meridians, stagnation of qi, and blood circulation for a long time. The treatment is mainly based on removing phlegm and softening the hard, promoting blood circulation, and clearing the meridians, supplemented by clearing away heat and detoxifying. Despite these treatments, surgical complications are unavoidable. Therefore, other methods are needed to assist surgical treatment [11].

To this end, preoperative embolization of tumors with abnormal blood supply is encouraged when necessary to reduce intraoperative bleeding and facilitate the surgery. Super-selective embolization of intratumoral vessels [12] refers to the delivery of a microcatheter into the blood supply artery of a meningioma patient, through which an embolic agent is injected to block the blood flow, prevent intraoperative bleeding, and soften the tumor, thereby reducing the difficulty of surgical resection and facilitating surgical resection [13, 14]. However, due to the paucity of related clinical studies, the clinical effectiveness of this procedure has not been fully clarified. In view of this, this study aims to evaluate the effectiveness of super-selective embolization for parasagittal meningiomas and its effect on the level of inflammatory factors, so as to provide clinical references for treatment.

## 2. Materials and Methods

### 2.1. Participants

A total of 48 patients with parasagittal meningiomas diagnosed and treated in our hospital from September 2018 to March 2020 were randomly included and assigned to receive meningioma resection (control group) or meningioma resection plus super-selective embolization (study group), with 24 patients in each group. The included patients were aged 22–75 years, with 19 males and 29 females. The randomization was carried out using an online web-based randomization tool (freely available at http://www.randomizer.org/). For concealment of allocation, the randomization procedure and assignment were managed by an independent research assistant who was not involved in the screening or evaluation of the participants.

This was a retrospective study supervised by the ethics committee of Cangzhou Central Hospital (No. ChiCTR2200077981) with no interference with the treatment process.

The original sample size calculation estimated that 24 patients in each group would be needed to detect a 3-point difference between groups in a two-sided significance test with a power of 0.8 and an alpha error level of 0.05.

### 2.2. Inclusion and Exclusion Criteria

Inclusion criteria: ① Patients who met the clinical diagnostic criteria and were diagnosed with parasagittal meningiomas by relevant imaging, with a tumor diameter of ≥ 5 cm, and who provided written informed consent were included. ② In line with the indications for surgery; ③ Positive by vascular ultrasound or intravenous contrast examination; ④ No severe cardiopulmonary failure, severe liver and kidney insufficiency, malignant tumor, and other diseases.

Exclusion criteria: ① Patients with endocrine disorders, coagulation disorders or hematologic disorders, or with relevant surgical contraindications were excluded. ② Discharge or death within 24 hours of admission; ③ Incomplete clinical medical records; a history of severe coagulation disorders and blood system-related diseases; ④ severe lower extremity deformities, arteriosclerosis, infectious diseases, and mental disorders.

### 2.3. Methods

Patients in the control group underwent meningioma resection. The surgical approach was determined based on a preoperative cranial CT scan. A unilateral craniotomy was performed with a bone flap reaching the midline of the head, and the dura mater was removed by electrocoagulation to reduce tumor blood flow. The tumor was first separated from the lateral wall of the superior sagittal buccal cavity and resected along the tumor-brain interface. The base of the tumor in the lateral wall of the superior sagittal sinus was subsequently cauterized, and the dura was repaired with periosteum or artificial membrane, followed by the closure of the skull [15].

Patients in the study group underwent meningioma resection preceded by super-selective embolization. The femoral artery was percutaneously punctured using the Seldinger technique followed by the placement of a 5F catheter. The enhanced contrast agent was then injected to monitor the donor artery, and a microcatheter was super-selectively inserted into the donor artery on fluoroscopy and embolized with polyvinyl alcohol pellets until the donor artery disappeared. one week after embolization, meningioma resection was then performed in the same manner as in the control group.

### 2.4. Evaluation Criteria

① Clinical indices: clinical surgery-related indices, including operative time and intraoperative bleeding, were recorded and compared in detail for both groups.

② Tumor resection outcome: Simpson grading [16] was used to assess the tumor resection after surgery in both groups.

③ Inflammatory factors: 5 ml of fasting venous blood was collected from the two groups of patients before and after treatment and centrifuged at 3000 r/min for 15 min to obtain the serum. Serum levels of interleukin-6 (IL-6), tumor necrosis factor-*α* (TNF-*α*), and hypersensitive C-reactive protein (hs-CRP) were measured by enzyme-linked immunosorbent assay and compared, and the kits were purchased from Nanjing Jiancheng Institute of Biological Engineering.

④ Postoperative follow-up: a three-month postoperative follow-up was performed by outpatient follow-up. Contrast-enhanced magnetic resonance imaging (MRI) was used to assess the presence of tumor recurrence, and the follow-up results of the two groups were compared.

### 2.5. Statistical Analysis

GraphPad Prism 8 software was used to visualize the data obtained in this study into matching images, and SPSS 22.0 software was used for data analyses. The measurement data were expressed as (mean ± standard deviation) and analyzed by an independent sample *t*-test. The count data were expressed as the number of cases (%) and analyzed by the chi-square test. Differences were suggested to be statistically significant at *P* < 0.05.

## 3. Results

### 3.1. Patient Characteristics

There were 24 patients in the control group, 10 males and 14 females, aged 22–73 (50.33 ± 6.12) years, with a maximum tumor diameter of 5.1–7.7 (5.84 ± 0.41) cm, the disease duration was (2.42 ± 0.79) years. 8 with an education level of high school or less, and 16 of undergraduate or above. In the study group, there were 24 patients, 9 males, and 15 females, aged 24–75 (50.42 ± 5.97) years, with a maximum tumor diameter of 5.0–7.6 (5.93 ± 0.37)cm, the disease duration was (2.14 ± 1.17) years. 7 with an education level of high school or less, and 17 of undergraduate or above. The patient characteristics of the two groups were comparable (*P* > 0.05). (Table 1).

### 3.2. Clinical Surgical Indicators

Patients in the study group had shorter operative time and less intraoperative bleeding (299.87 ± 25.96, 315.69 ± 81.04) compared to patients in the control group (365.21 ± 39.87, 472.52 ± 105.59) (*P* < 0.05). (Table 2).

### 3.3. Tumor Resection Outcome

The study group had more patients with Simpson I resection (87.50%) than the control group (62.50%) (*P* < 0.05). (Figure 1).

### 3.4. Inflammatory Factors

There was no statistically significant difference in the inflammatory factor levels between the two groups of patients before treatment (*P* > 0.05). After treatment, the levels of IL-6, TNF-*α*, and hs-CRP in patients in the study group (80.45 ± 24.01, 132.54 ± 40.69, and 12.21 ± 1.07) were lower than those in patients in the control group (104.25 ± 23.62, 189.55 ± 43.58, and 20.17 ± 1.55) (*P* < 0.05). (Table 3).

### 3.5. Postoperative Follow-Up

The results of the three-month follow-up showed that one patient in the study group was reoperated for tumor recurrence and no patient died, while three patients in the control group were reoperated for tumor recurrence and one patient died. The difference in recurrence and mortality rate between the two groups was not statistically significant (*P* > 0.05). (Table 4).

## 4. Discussion

Meningiomas are one of the most common intracranial tumors, most of which occur in the sagittal sinus of the cerebral hemisphere. Meningiomas form the pedicle of the tumor by adhering to the dura mater, and the blood of the external carotid artery can supply blood to the tumor through this pedicle. Therefore, the blood circulation at the site of meningioma is rich, which makes the surrounding skull easily eroded, resulting in skull hyperplasia, tortuous and inflamed scalp veins, and in severe cases, skull necrosis or skull defect may occur. Parasagittal meningiomas grow slowly, and the early symptoms are not obvious. When patients have epilepsy, headache, or even hemiplegia or dementia, their intracranial mass is more obvious [17]. Compression of the tumor results in obstruction of the corresponding venous return, leading to the possibility of intracranial hypertension in the patient. Large parasagittal meningiomas have special growth sites and large tumor diameters, making it difficult to completely resection them, so they have a higher recurrence rate than other sites [18].

Meningiomas can be classified as “brain tumors” in traditional Chinese medicine. “Lingshu·All Diseases Beginning” states “The blood coagulation accumulates in but does not disperse, and the body fluid is astringent and seeps, and it does not go away, and it accumulates.” The main pathogenesis of brain tumors is wind, phlegm, toxin, blood stasis, and deficiency, which is based on the loss of liver and kidney, phlegm turbidity obstructs the orifices, and poison and blood stasis are the targets. Physicians of the past dynasties have different opinions on the syndrome differentiation and treatment of the etiology and pathogenesis of brain tumors [19, 20]. Although Chinese medicine also has good effects, it is mostly used for postoperative recovery. Therefore, it is particularly important to improve the therapeutic effect of surgery.

Preoperative tumor embolization has become an important routine adjunct for intracranial high blood flow tumors, especially meningiomas [21] The expected outcome is complete occlusion of the tumor vascular system to induce ischemia, necrosis, and atrophy of the tumor, thereby facilitating its isolation from the surrounding tissue, reducing intraoperative bleeding, shortening operative time, improving tumor resection rate, and avoiding surgical complications. However, in conventional preoperative embolization, the embolization catheter can only reach the branch entrance of the external carotid artery, which suggests a high risk of surgical errors and may cause complications such as severe hemiparesis, aphasia, and coma. [22]. Super-selective embolization uses a microcatheter to avoid other normal arteries and protect the main trunk and major branches of the external carotid artery to reduce the incidence of complications such as local skin pain, numbness, fever, scalp necrosis, misembolization, and even cerebral infarction [23, 24]. Herein, 48 patients with parasagittal meningiomas were included in this study to evaluate the effectiveness of super-selective embolization for parasagittal meningiomas and its effect on the level of inflammatory factors.

The results of this study showed that super-selective embolization prior to meningioma resection achieved shorter operative time and less intraoperative bleeding, suggesting that super-selective embolization treatment was effective in controlling intraoperative bleeding and reducing the difficulty of surgery versus single meningioma resection. The explanation for this might be that meningioma angiography clarifies the diagnosis, establishes blood flow and anatomical position of the tumor, and improves the creation and implementation of the surgical plan. Selective embolization cuts off the blood supply to the tumor, minimizing bleeding while guaranteeing an unobstructed operational field and optimum tumor excision. Clinical studies have shown that the use of super-selective embolization for parasagittal meningiomas enables more complete resection of the lesion, prevents blood circulation to the meningioma [25], and boosts postoperative recovery, which is similar to the results of the present study. Here, the study group had more patients with Simpson I resection (87.50%) than the control group (62.50%). Previous studies suggest that if the superior sagittal buccal cavity is patent, Simpson grade II resection is available to avoid serious consequences such as venous cerebral infarction, cerebral hemorrhage, or death due to superior sagittal buccal lesions; if the tumor causes complete occlusion of the superior sagittal buccal cavity, the superior sagittal buccal cavity can be resected anatomically from the occlusion site to achieve Simpson I resection [26] The results of the current study suggest that preoperative super-selective embolization facilitates the successful implementation of Simpson I resection of tumors. The inflammatory response has been reported to be associated with tumor tissue infiltration. The tumor stroma contains tumor-associated macrophages that induce immune responses in the body and stimulates the growth of tumor cells. Herein, the levels of IL-6, TNF-*α*, and hs-CRP in the study group were lower than those in the control group after treatment, suggesting that super-selective embolization for patients with parasagittal meningiomas could reduce the inflammatory response and avoid disease deterioration to ensure long-term efficacy. Hs-CRP is an acute-phase protein synthesized by the liver that sensitively reflects the magnitude of the inflammatory response, and TNF-*α* is an inflammatory reaction initiator that causes inflammatory damage and promotes the inflammatory response and the release of proinflammatory factors such as IL-6, and the proliferation of activated T cells further intensifies the inflammatory response. The results of this study are consistent with the findings of Vivian et al. which showed that super-selective embolization plus resection of meningioma reduced surgical trauma and inflammatory response and ameliorated the prognosis of patients. Furthermore, the results of the three-month follow-up showed that one patient in the study group was reoperated due to tumor recurrence and no patient died, while three patients in the control group were reoperated due to tumor recurrence and one patient died. However, the difference in recurrence and mortality rate between the two groups did not come up to the statistical standard (*P* > 0.05). The reason may be that compared with traditional surgery, super-selective embolization has a clear surgical field and can fully expose intracranial blood vessels, nerves, and tumors. The important brain tissue can greatly improve the success rate of surgery and reduce the occurrence of postoperative complications and recurrence.

This finding might be attributed to the study's small sample size and short follow-up period, as well as the distribution of tumor pathology types in both groups. To give more accurate results, future research with bigger sample size and long-term follow-up will be done.

## 5. Conclusion

The use of super-selective embolization for parasagittal meningiomas contributes to reducing intraoperative bleeding, effectively improving tumor resection and surgical safety, and lowering inflammatory factor levels. Further trials are, however, required before clinical promotion.

## Figures and Tables

**Figure 1:** Tumor resection outcome.

**Table 1:** Patient characteristics ($\bar{\text{x}}$ ±*s*).

Group	n	Gender		Age (years)		Maximum diameter of tumor (cm)		Education level	
		Male	Women	Scope	Average	Scope	Average	High schooland below	Undergraduateand above
Control group	24	10	14	22–73	50.33 ± 6.12	5.1–7.7	5.84 ± 0.41	8	16
Study group	24	9	15	24–75	50.42 ± 5.97	5.0–7.6	5.93 ± 0.37	7	17
*t-value*	—	—	—	—	0.052	—	0.798	—	—
*P-value*	—	—	—	—	0.959	—	0.429	—	—

**Table 2:** Clinical surgical indicators ($\bar{\text{x}}$ ±*s*).

Group	N	Operative time (min)	Intraoperative bleeding volume (ml)
Control group	24	365.21 ± 39.87	472.52 ± 105.59
Study group	24	299.87 ± 25.96	315.69 ± 81.04
*T value*	—	6.728	5.772
*P value*	—	<0.001	<0.001

**Table 3:** Levels of inflammatory factors ($\bar{\text{x}}$ ±*s*).

Time point	Inflammatory factors	Control group (*n* = 24)	Study group (*n* = 24)	*t-value*	*P -value*
Before treatment	IL-6 (pg/mL)	58.96 ± 10.24	59.23 ± 10.31	0.091	0.928
	TNF-*α* (pg/mL)	80.16 ± 11.54	80.33 ± 10.94	0.052	0.959
	hs-CRP (mg/L)	6.15 ± 1.21	6.16 ± 1.05	0.031	0.975

After treatment	IL-6 (pg/mL)	104.25 ± 23.62	80.45 ± 24.01	3.462	0.001
	TNF-*α* (pg/mL)	189.55 ± 43.58	132.54 ± 40.69	4.684	<0.001
	hs-CRP (mg/L)	20.17 ± 1.55	12.21 ± 1.07	20.704	<0.001

**Table 4:** Postoperative follow-up (%).

Group	n	Recurrence	Mortality
Control group	24	3 (12.50)	1 (4.17)
Study group	24	1 (4.17)	0 (0.00)
*x * ^*2*^	—	1.091	1.021
*P-value*	—	0.296	0.312

## Data Availability

All data generated or analyzed during this study are included in this published article.
